RETRACTED

# Sodium nitroprusside application improves morphological and physiological attributes of soybean (*Glycine max* L.) under salinity stress

**DOI:** 10.1371/journal.pone.0248207

**Published:** 2021-04-16

**Authors:** Zahra Jabeen, Hafiza Asma Fayyaz, Faiza Irshad, Nazim Hussain, Muhammad Nadeem Hassan, Junying Li, Sidra Rehman, Waseem Haider, Humaira Yasmin, Saqib Mumtaz, Syed Asad Hussain Bukhari, Ahlam Khalofah, Rahmah N. Al-Qthanin, Moodi Saham Alsubeie

**Affiliations:** 1 Department of Biosciences, COMSATS University Islamabad (CUI), Islamabad, Pakistan; 2 Institute of Crop Science, Zhejiang Key Laboratory of Crop Germplasm, Zhejiang University, Hangzhou, PR China; 3 Bio-Ultrastructure Analysis Laboratory of Analysis Center of Agrobiology and Environmental Sciences, Zhejiang University, Hangzhou, PR China; 4 Department of Agronomy, Bahauddin Zakariya University, Multan, Pakistan; 5 Department of Biology, Faculty of Science, King Khalid University, Abha, Saudi Arabia; 6 Research Center for Advanced Materials Science (RCAMS), King Khalid University, Abha, Saudi Arabia; 7 Prince Sultan Bin-Abdul-Aziz Center for Environment and Tourism Studies and Researches, King Khalid University, Abha, Saudi Arabia; 8 Biology Department, College of Sciences, Imam Mohammad Ibn Saud Islamic University, Riyadh, Kingdom of Saudi Arabia; Harran Üniversitesi: Harran Universitesi, TURKEY

## Abstract

Salinity is among the major abiotic stresses negatively affecting the growth and productivity of crop plants. Sodium nitroprusside (SNP) -an external nitric oxide (NO) donor- has been found effective to impart salinity tolerance to plants. Soybean (*Glycine max* L.) is widely cultivated around the world; however, salinity stress hampers its growth and productivity. Therefore, the current study evaluated the role of SNP in improving morphological, physiological and biochemical attributes of soybean under salinity stress. Data relating to biomass, chlorophyll and malondialdehyde (MDA) contents, activities of various antioxidant enzymes, ion content and ultrastructural analysis were collected. The SNP application ameliorated the negative effects of salinity stress to significant extent by regulating antioxidant mechanism. Root and shoot length, fresh and dry weight, chlorophyll contents, activities of various antioxidant enzymes, i.e., catalase (CAT), superoxide dismutase (SOD), peroxidase (POD) and ascorbate peroxidase (APX) were improved with SNP application under salinity stress compared to control treatment. Similarly, plants treated with SNP observed less damage to cell organelles of roots and leaves under salinity stress. The results revealed pivotal functions of SNP in salinity tolerance of soybean, including cell wall repair, sequestration of sodium ion in the vacuole and maintenance of normal chloroplasts with no swelling of thylakoids. Minor distortions of cell membrane and large number of starch grains indicates an increase in the photosynthetic activity. Therefore, SNP can be used as a regulator to improve the salinity tolerance of soybean in salt affected soils.

RETRACTED

## Introduction

Soybean is an important legume crop grown around the world for its edible beans. Soybean demand is hiking around the world due to its unique seed composition and excellent nutritional value [1]. Soybean seeds contain high amount of protein and oil with no cholesterol [2]. Soybean is cultivated under different environments; however, susceptibility of the crop to various biotic and abiotic stresses negatively impacts its productivity [3]. More specifically, soybean is sensitive to salinity stress compared with other major crops, i.e., rice, cotton and wheat. Salinity stress hinders germination, nodule generation, plant development and seed yield of soybean [4]. Soil salinity is a serious problem in irrigated areas, as it decreases yield and quality of the crops grown on salt-affected silos [5]. Osmotic stress and ionization toxicity are among the initial negative impacts posed by salinity to crop plants [6]. However, the plants have evolved a variety of defense mechanisms by restructuring physiology, biochemistry and molecular machinery to reduce nutrient imbalance and oxidative stress caused by reactive oxygen species (ROS) accumulation, such as H_2_O_2_ and O_2_^-^ under salinity stress [7, 8]. Sodium (Na^+^) is a common soluble ion in soil that is harmful to the majority of crop plants. The Na^+^ ion is not necessary for the growth of most of the plants; thus, excessive Na^+^ accumulation in cells disturbs osmotic, oxidative and ionic homeostasis [9, 10]. Therefore, prevention of Na^+^ accumulation and maintenance of appropriate K^+^/Na^+^ ratio in cytoplasm are important for growth and survival under salinity stress [11, 12].

The ROS causes significant damage to the membrane and other cellular structures of soybean under salinity stress. The ability of ROS to interact with many cellular components inhibits plant growth [13]. Plants stimulate intracellular defense system by inducing ROS scavenging enzymatic and non-enzymatic antioxidants, such as catalase (CAT), superoxide dismutase (SOD), peroxidase (POD) and ascorbate peroxidase (APX) to eliminate the toxic molecules to cope with salinity stress [14–16].

Nitric oxide (NO) is multitasking signaling molecule and involved in stress-acclimation processes of plants. The NO plays a pivotal role in plant developmental processes, including seed germination, plant development, photosynthesis, stomatal movement, recovery of cell membrane etc. [17, 18]. Moreover, SNP is demonstrated as one of the important components of plant responses to abiotic and biotic stresses [19–21].

RETRACTED

The use of SNP to improve stress tolerance of crop plants has been recently increased. However, physiological and biochemical roles of SNP in salinity tolerance are still unclear. Nonetheless, almost no study has been conducted to infer the role of SNP in improving salinity tolerance of soybean. Therefore, current study was aimed at inferring the role of exogenous application of SNP in improving salinity tolerance of soybean. It was hypothesized that exogenous SNP application will improve morphological, physiological and biochemical attributes of soybean under salinity stress. Furthermore, SNP-induced increased activities of various antioxidant enzymes will help soybean to better tolerate salinity than no application of SNP. The results will help to improve soybean growth and productivity in salt-affected regions of the world.

## Materials and methods

### Plant material and hydroponic culture technique

The seeds of a widely cultivated soybean genotype NARC-2 were obtained from National Agriculture Research Center (NARC) Islamabad, Pakistan. Seeds were surface sterilized in 3% sodium hypochlorite solution for 10 min, and washed thrice with distilled water. Afterwards, seeds were sown in germination trays. Seedlings were grown at room temperature (25°C to 30°C) with 8 h dark and 16 h light period. Uniform seedlings were transferred from germination trays to hydroponic nutrient solution (half-strength pH:5.5–6) after 7 days of germination. The one-liter plastic pots containing seedlings were placed in glass house adjusted with 16 h photoperiod, 30/35 day/night temperature and 75% relative humidity. After one week, plants were treated with full-strength Hoagland nutrient solution. Nutrient solution was refreshed every week for one month. The nutrient solution was prepared according to Zahra et al. [22]. After one month, NaCl and SNP treatments were initiated and each treatment had three replications. Four-weeks-old seedlings were treated under 4 different treatments, i.e., T_1_-control (0 mM NaCl + 0 μM SNP), T_2_-NaCl stress and SNP (100 mM NaCl + 10 μM SNP), T_3_-SNP alone (10 μM SNP) and T_4_-NaCl stress alone (100 mM NaCl). The experiment was arranged as a completely randomized design (CRD). Plants were harvested four weeks after the initiation of treatment to evaluate the effects of salinity stress.

### Growth traits

The length of root, shoot and whole plant was measured from all plants and averaged. Fresh weight (FW) of root, shoot and whole plant from each treatment was recorded on an electronic balance and then these samples were dried in an oven for 72 h at 70°C. Dry weight of the root, shoot and plant samples was then recorded to measure dry weight.

RETRACTED

### Chlorophyll contents

Chlorophyll contents were measured according to Gitelson et al. [23]. Briefly, fresh leaves were detached from the plants and chopped. Afterwards 10 ml of dimethyl sulfoxide (DMSO) was added to 0.05 g leaf samples. The resulting mixture was incubated at 65°C for 72 h in water bath. The extract obtained after incubation was centrifuged for 5–10 min at 7000 rpm and supernatant was collected. The supernatant was then read at 663 nm, 645 nm, and 480 nm wavelengths for determination of chlorophyll-a, chlorophyll-b and carotenoid, respectively.

### Estimation of lipid peroxidation/MDA content

The MDA content/lipid peroxidation was assayed by measuring malendialdehyde according to the procedure described by Esfandiari et al. [24]. Plant samples were mixed in 2.5 ml of 5% trichloroacetic acid (TCA) and thiobarbitaric acid and 1.5 ml of crude enzyme extract. The homogenate was heated at 95°C for 15 min, chilled on ice and mixture was centrifuged at 4800 rpm for 10 min. Supernatant was collected and wavelength was recorded at 532 nm by deducting the non-specific absorption at 600 nm.

### Antioxidant enzyme extraction and assay

Enzymes were extracted according to the method of Esfandiari et al. [24]. For SOD, CAT, APX, POD, PPO, PAL and MDA extraction, 0.5 g of leaf and 0.3 g of root samples were ground in chilled 0.1 M phosphate buffer solution (pH 7.5) with pre-chilled mortar and pestle. Extract from each treatment were centrifuged at 8000 rpm and 4°C for 20 min. Supernatant was collected for enzyme assays.

The SOD activity was determined according to Kumar et al. [25] through measuring nitroblue tetrazolium (NBT) inhibition in photo-reduction. The extract contained 5 μM riboflavin, 18.75 μM NBT, 32 mML-methionine and 25 μM EDTA in 250 ml distilled water. Reaction mixture contained 2.75 ml of reaction solution, 0.25 ml of d.H_2_O + 0.025 ml of enzyme extract. The SOD reaction was carried out under light of 4000 flux at room temperature for 20 min. Wavelength was recorded after 20 min at 560 nm using spectrophotometer. The CAT activity was measured by following Kumar et al. [25]. The solution mixture contained 50 mM sodium phosphate buffer solution (pH 7.0), 0.1 ml enzyme extract, 300 mM H_2_O_2_ and 0.1 ml deionized water. Wavelength was observed at 240 nm. The POD activity was measured according to the method of Kumar et al. [25]. The reaction mixture contained 0.5 ml 1% H_2_O_2_, 1.5 ml 0.05 M pyrogallal phosphate buffer (pH 6.8). Solution was incubated for 10 min at room temperature. Absorbance was recorded at 436 nm. The APX activity was estimated by following Siddiq and Dolan [26]. The reaction mixture contained 0.1 ml 7.5 mM ascorbic acid (ASA), 0.1 ml 300 mM H_2_O_2_, 2.7 ml 50 mM phosphate buffer (pH 7.0) and 0.1 ml enzyme extract. Wavelength was observed at 290 nm. Siddiq and Dolan [26] were followed to measure PPO activity. Reaction solution contained 1.5 ml 0.1 M sodium phosphate buffer (pH 6.5), 0.2 ml crude enzyme extract and 0.2 ml 0.01 M of chatechole. Afterwards, reading was measured at 495 nm. Gao et al. [27] were followed to measure PAL activity. Solution mixture contained 0.03 ml 150 mM of tris-HCL, 0.03 ml crude enzyme extract and 0.67 ml 3 mM L-phenylalanine. Wavelength was measured at 270 nm.

RETRACTED

### Determination of Na and K ions

The Na and K ions were measured according to Pii et al. [28]. Leaf and root samples were dried at 80°C and ground to fine powder by using grinding mill. A measured quantity of resulting powder was added 10 ml nitric acid and perchloric acid inside fume hood. The mixture was boiled on hot plate at 150–235°C following overnight incubation at room temperature until the formation of fumes. Then mixture was cooled for 2–4 min and rinsed with 3 ml distilled water. Samples were diluted with distilled water up to 50 ml. After filtration with Whatman paper, Na^+^ and K^+^ contents were estimated with a Shimadzu AA-680 atomic absorption flame spectrophotometer.

### Transmission electron microscopy (TEM)

For TEM, fresh root tip samples and leaf fragments were fixed in 2.5% glutaraldehyde for 3h, washed five times with 0.1 M sodium phosphate buffer (pH 7.0) and fixed into 1% OsO_4_ for 1 h. The samples were then completely desiccated in a series of ethanol (30 to 100%) and acetone, and processed further according to Zahra et al. [29].

### Statistical analysis

The collected data were tested for normality using Shapiro-Wilk normality test, which indicated a normal distribution. Therefore, original data were used in statistical analysis. One-way analysis of variance (ANOVA) was used to test significance in the data. Least significant difference (LSD) test at 5% probability was used to separate means where ANOVA indicated significant differences. All statistical computations were executed on Statistix 8.1 software. The data were presented as means ± standard errors of means (SE).

## Results

### Growth traits

Salinity stress caused a significant decrease in root, shoot and whole plant biomass compared to control treatment. The reduction in in root, shoot and whole plant biomass was 40%, 46% and 52%, respectively compared with control (S1 Table in S1 File). SNP application lowered the reduction in these traits and it was reduced to 12%, 14% and 21% with 0 μM SNP application under salinity stress (S1 Table in S1 File). Salinity stress also decreased fresh and dry weight of shoot, root and whole plant (S2 Table in S1 File). Fresh weight of root, shoot and whole plant was reduced by 46%, 38% and 56%, respectively under salinity stress compared with control treatment. Similarly, a reduction of 48%, 33% and 34% was recorded in dry weight of root, shoot and whole plant, respectively under 100 mM salinity (S2 Table in S1 File). However, 10 μM SNP application increased root, shoot and whole plant fresh and dry weight by 38%, 29%, 75% and 58%, 27% and 29%, respectively compared to no SNP application under salinity stress (S2 Table in S1 File).

RETRACTED

### Chlorophyll and MDA contents

Salinity stress adversely affected cell membrane integrity as an increase was observed in membrane injury. Exogenous application of 10 μM SNP tended to repair detrimental effect of salinity stress. Leaf and root MDA contents were increased by 38% and 44%, respectively under salinity stress compared with control treatment (Fig 1A–1D). Nonetheless, SNP application under salinity stress caused less damage to shoot (16%) and root (10%) as compared to no SNP application.

**Fig 1:** Analysis of MDA content in leaves and roots (a, b) and chlorophyll contents (c, d) of treated and control plants of soybean. Data are means ± SD calculated from three replicates.

Salinity stress caused a significant decrease in chlorophyll-a and b contents compared to control treatment. A reduction of 48% and 58% was recorded in chlorophyll-a and b, respectively (Fig 1C and 1D). However, exogenous application of SNP under salinity stress increased total chlorophyll contents compared to no SNP application. Increased chlorophyll-a (38%), and chlorophyll-b (44%) contents were observed with SNP application under salinity compared to salinity alone (Fig 1C and 1D).

### Activities of antioxidants enzymes

The SOD activity was increased in root and leaf tissues under salinity stress compared with control. The SOD activity was increased by 67% and 45% in leaf and root, respectively under 100 mM salinity stress relative to 0 mM salinity (Fig 2). Exogenous SNP application increased SOD activity 40% and 79% in leaf and root, respectively under salinity stress relative no SNP application under salinity (Fig 2A and 2B).

**Fig 2:** Activities of SOD, CAT and POD content in leaves (a, c, e) and roots (b, d, f) of treated and control soybean plant. Data are means ± SD calculated from three replicates.

RETRACTED

The CAT activity was increased by 60% and 37% in leaves and roots respectively under salinity stress as compared with control (Fig 2C and 2D). The SNP application under salinity increased CAT activity by 32% and 62% in leaves and roots compared with no SNP application (Fig 2C and 2D). A significant increase in POD activity was recorded under salinity stress compared to control treatment (Fig 2E and 2F). An increase of 228% in POD activity of leaf and 44% in root was observed under 100 mM salinity compared with no salinity. Exogenous application of SNP under salinity proved beneficial as it increased POD activity by 444% and 71% compared with no SNP application under 100 mM salinity stress (Fig 2E and 2F). The APX activity was increased by 6% and 129%, respectively in roots and leaves under 100 mM salinity stress relative to non-saline control (Fig 3A and 3B). The PPO activity was increased by 28% and 57% in both leaf and root under 100 mM salinity compared to control (Fig 3C and 3D). The SNP application elevated PPO activity by 42% and 103% in leaf and root, respectively under 100 mM salinity compared with no application of SNP under salinity (Fig 3C and 3D). Activity PAL was significantly higher in leaves and roots under salinity relative to control (Fig 3E and 3F). Exogenous application of SNP induced more increase in PAL activity under 100 mM salinity compared with no SNP application (Fig 3E and 3F).

**Fig 3:** Activities of APX, PPO and PAL content in leaves (a, c, e) and roots (b, d, f) of treated and control soybean plant. Data are means ± SD calculated from three replicates.

### Na^+^ and K^+^ ion contents

High Na^+^ contents along with lower K^+^/Na^+^ ratio were recorded under salinity stress. The Na^+^ content was increased by 285% and 212%, whereas, K^+^ content was decreased by 39% and 43% in leaf and root, respectively, compared with salinity-free treatment (Table 1). Exogenous application of SNP resulted in lesser accumulation of Na^+^ content in leaf (117%) and root (119%) whereas, 15% decrease in K^+^ content in leaf and 18% in root was observed as compared to no SNP application (Table 1).

**Table 1:** Effect of different salinity and exogenous SNP application treatments on Na^+^ (ppm) and K^+^ (ppm) accumulation and Na^+^/Ka^+^ ratio.

Treatments	Leaf Na^+^	Root Na^+^	Leaf K^+^	Root K^+^	Leaf Na^+^/K^+^	Root Na^+^/K^+^
0 mM salinity	35±6.8^c^	41±9.1^d^	159±2.8^b^	115±2.7^b^	0.21±0.005^c^	0.35±0.07^c^
SNP with no salinity	30.0±2.9^c^	53±3.6^c^	130±4.9^a^	130±4.9^a^	0.17±0.018^c^	0.41±0.01^c^
100 mM salinity	135±4.5^a^	128±6.8^a^	65±4.2^d^	65±4.2^d^	1.20±0.058^a^	1.31±0.07^a^
100 mM salinity + SNP	76.7±9.3^b^	90±8.4^b^	94±7.0^c^	94±7.0^c^	0.56±0.04^b^	1.07±0.01^b^

Values presented are the mean ± SD (n = 3). Means followed by different letters on values show statistically significant differences at P ≤0.05.

RETRACTED

A strong positive correlation was noted among activities of antioxidant enzymes such as SOD, APX, CAT, POD and PAL, whereas MDA content had negative correlation with root length, fresh and dry weight, chlorophyll a, chlorophyll b and shoot length (Fig 4A and 4B).

**Fig 4:** Correlation matrix of (a) root and (b) leave of biochemical and physiological traits of different treatments. The name of the parameters was presented on diagonal line. The upper side of the figure depicted correlation coefficient and the lower side of figure showed the bivariate.

### Ultrastructure of mesophyll, chloroplast and root cells

Chloroplast and mesophyll cells SNP-treated plants showed normal ultrastructure with few plastoglobules, small starch grains with compactly arranged thylakoids and well-organized grana stacks containing well-developed outer envelope. Mesophyll cell membrane was in close contact with cell wall. Moreover, increased number of chloroplasts per mesophyll cell was observed in control and SNP-treated plants under non-saline condition relative to salt stressed plants (Fig 5A, 5B, 5D and 5E). However, plants grown under 100 mM salinity showed obvious ultrastructural changes including, swellings of chloroplast, disintegrated plasma membrane envelope, dissolved thylakoids with reduced grana stacking and few plastoglobuli, as compared to control and co-application of SNP under salinity stress. Moreover, salinity alone resulted in disintegration of mesophyll cell, chloroplasts and cell membrane (Fig 5G and 5H). Application of SNP under salinity stress showed slight alterations in cell organelles (Fig 5G and 5K) as compared to no SNP application. The alterations included slightly oval shaped chloroplast with closely packed grana thylakoids similar to control plants. Moreover, fewer plastoglobuli, and large number of starch grains were observed (Fig 5G and 5K). The root cells of control and SNP treated plants under salinity-free treatment (Fig 5C and 5D) showed rich cytoplasm and well-developed cell organelles with smaller vacuoles and large and round nucleus. More number of plastoglobuli were observed in SNP-treated plants under no salinity. Salinity stress without SNP application showed fatal injury to the root cells, as the area of degraded cell organelles was wider with distorted cell shape, abnormal nucleus structure, disrupted nucleolus and shrunken vacuole compared to the plants treated with SNP under salinity stress (Fig 5I). The SNP application under salinity stress prevented root cells from injures as cell organelles were apparently similar to control plants (Fig 5L).

RETRACTED

**Fig 5:** Transmission electron micrographs of chloroplast (a, d, g, j), mesophyll cells (b, e, h, k) and root (c, f, i, l) of control and treated plants. Bar = 0.5μm, 1μm and 2μm.

## Discussion

Salinity stress negatively influenced the morphological, physiological and biochemical attributes of soybean under salinity stress. Exogenous application of SNP, as hypothesized, improved morphological, physiological and biochemical attributes of soybean under salinity stress. Esim and Atici [30] reported that SNP is a prime signaling molecule capable of improving growth and physiological function of plants under a variety of abiotic and biotic stresses. This study revealed that salinity stress hampered biomass production and growth of soybean. Similar negative impacts of salinity has been observed in several crops, including tomato [31], rice [32], maize [33], barley [34] and wheat [35]. The SNP application (10 μM) significantly improved biomass of salt-stressed plants in the current study, which are in line with the earlier report of Tian et al. [36] for wheat crop. However, it is reported that SNP application can reduce solute potential, while elevates water potential under osmotic stress [37], which could be a plausible reason for increasing soybean biomass in the current study. A reduction was observed in plant biomass and growth under salinity stress, which could be attributed to inhibition of plant growth due to oxidative damage to cells under unavailability of water [37–39].

Our study revealed that salt stress affected chloroplast structure and decreased chlorophyll content resulting in reduced photosynthesis. Moreover, decreased photosynthesis rate can be attributed to disturbed activities of the enzymes involved in chlorophyll biosynthesis, stomatal conductance and intercellular CO_2_ concentration [15, 40]. However, decrease in chlorophyll contents was significantly improved by SNP application, which may be due to the inhibition of ROS production or sustaining the stability of photosynthetic mechanism [36]. The results of the current study are in line with those of Muthulakshmi et al. [41], who indicated that SNP application could improve chlorophyll contents, transpiration rate and photosynthetic efficiency under salinity stress. The SNP application under salinity stress improved photosynthetic pigments by protecting cell membrane organelle containing chlorophyll against salinity-induced ion toxicity [42, 43].

The roots and leaves accumulated higher MDA content thereby increasing electrolyte leakage. Kaya et al. [44] suggested that increased MDA content are owed to membrane destruction due to oxidative damage. The SNP application decreased MDA content and electrolyte leakage under salt stress, which is in accordance with the previous observations [45, 46]. Consequently, SNP application can be an effective way to prevent plants from oxidative damage under salinity stress [47–49].

RETRACTED

Increased activities of CAT, SOD, APX, POD, PAL and PPO were observed under salinity stress. Similar findings of increased activities of these enzymes are reported by Manai et al. [50] in *S*. *lycopersicum*. Bai et al. [51] reported that antioxidant enzymes are generally known as ROS scavengers in plants under salinity stress. Moreover, SNP application under salinity stress increased the activities of CAT, SOD, APX, POD, PAL and PPO, which is in accordance with prior findings reported for rice crop [19, 52]. Application of SNP may stimulate gene expression associated with antioxidant enzymes that could help plants to withstand salinity stress [38, 53].

Mohsenzadeh and Zohrabi [54] reported that SNP could increase POD, SOD, APX and CAT activities by mitigating the damage and enhancing the capability of scavenging radicals along with reduced MDA contents [55–58]. Moreover, our study revealed that salinity stress elevated Na^+^ content and reduced K^+^ content in the roots and leaves of soybean plants. High Na^+^ content disrupts Na^+^/K^+^ ratio, which may be due to increased Na^+^ influx [59, 60]. Ji et al. [60] suggested that decreasing K^+^ and increasing Na^+^ contents might be due to competition between K^+^ and Na^+^ ion absorption by plant roots. Increased Na^+^ accumulation results in higher Na^+^/K^+^, which distorts ion homeostasis by reducing Mn, Zn, and Mg contents. The SNP application under salinity stress increased K^+^ and decreased Na^+^ contents. Dong et al. [61] reported that SNP application under salinity stress could increase absorption of K^+,^ Mg^2+^, Ca^2+^ ions and decreases Na^+^ content, which might be attributed to the fact that SNP restricts uptake of Na ions into plant tissues. The mitigating effect of SNP under salt stress was also observed via transmission electron microscopy in the current study. Chloroplast and mesophyll cells of salinity-free and SNP application under no salinity treatments showed normal chloroplast ultrastructure with no obvious changes, while swelling of thylakoids, distortions of grana stacks under salt stress were due to change in element contents of stroma, destruction of photosynthetic apparatus, leaf senescence and ion toxicity [62, 63]. In present study SNP application under salt stress played a protective role in maintaining normal chloroplasts with no swelling of thylakoids, minor distortions of cell membrane and large number of starch grains. This resulted in increased photosynthetic activity, appropriate regulation of osmolytes and reduce Na^+^ ion toxicity, which have also been reported in earlier studies [2, 29, 64]. Root cell damage under salinity stress was mainly due to failure of water absorption, Na^+^ and Cl^-^ ions compartmentalization in vacuole due to decreased cell wall turgidity and reduced vacuole size as reported in earlier studies [22, 65, 66]. It is also well-known that higher number of plastoglobuli under salt stress is attributed to membrane breakdown [67]. However, we observed that SNP application under salinity stress prevented root cells from injures. The SNP plays a pivotal role in terms of root and cell wall repair, less membrane damage, and/or sequestration of Na^+^ ion in the vacuole, which is typically associated with the enhancement of antioxidant defense systems [66].

RETRACTED

## Conclusion

Salinity stress posed negative impacts on growth and physiological attributes and activities of antioxidant enzymes. Nonetheless, SNP application ameliorated the adverse effects of salinity by increasing activities of antioxidant enzymes. Based on results, it is concluded that SNP could play a vital role in elevating the antioxidant enzymes activity in response to salinity stress. Thus, the toxic effects of salinity were partially be eliminated by the exogenous application of SNP. Therefore, SNP could be used to improve growth and productivity of soybean crop in salt-affected soils.

## Supporting information

S1 File (DOCX)
